# Application of Reinforcement Learning Algorithm Model in Gas Path Fault Intelligent Diagnosis of Gas Turbine

**DOI:** 10.1155/2021/3897077

**Published:** 2021-09-17

**Authors:** Yulong Luo

**Affiliations:** School of Robot Engineering, Yangtze Normal University, Chongqing 408100, China

## Abstract

Gas turbine is widely used because of its advantages of fast start and stop, no pollution, and high thermal efficiency. However, the working environment of high temperature, high pressure, and high speed makes the gas turbine prone to failure. The traditional gas path fault intelligent diagnosis scheme of the gas turbine has the problems of poor control effect and low scheduling accuracy. Experiment studies the application of neural network and reinforcement learning algorithm in gas path fault intelligent diagnosis of the gas turbine. The accurate control of fault diagnosis planning is realized from gas path fault diagnosis, daily maintenance, service condition monitoring, power utilization rate, and other aspects of the gas turbine. The reinforcement learning model can realize the intelligent diagnosis and record of gas path fault of the gas turbine, to achieve diversified analysis and intelligent diagnosis scheme. Through neural network algorithm and deep learning technology, the whole process monitoring of the gas turbine is realized, and the failure rate of the gas turbine in the working process is reduced. The experimental results show that, compared with the thermal fault diagnosis method and the fault diagnosis method of the electric percussion drill, using thermal imaging, the gas turbine gas path fault intelligent diagnosis model based on the reinforcement learning algorithm can complete the data information in the process of real-time data transmission. The quantified conversion and processing of the system has the advantages of higher control accuracy and faster response speed, which can effectively improve the diagnostic efficiency and accuracy.

## 1. Introduction

At present, there are problems of poor reliability and low efficiency in the scheme of the gas turbine. The main reason is that the new generation of intelligent technology represented by deep learning is less applied [1]. Modern Internet technology and adaptive reinforcement learning technology had rapid development and construction, and the rapid development of data mining technology has also led to the reform of the gas turbine fault intelligent diagnosis scheme [2]. These technologies improve the application of intelligent gas path fault diagnosis scheme of the gas turbine. Therefore, intelligence and accuracy have become an important indicator of the advanced level [3]. How to establish an efficient and intelligent gas path fault intelligent diagnosis system of the gas turbine has become an important development direction in the process of gas turbine diagnosis [4]. At present, although the gas turbine diagnosis and control system, there are some problems in the query efficiency of diagnosis data and automatic control, such as slow control [5]. Moreover, it is difficult to analyze the detailed fault diagnosis control process [6]. Up to now, scholars still have some problems in gas path fault diagnosis of gas turbine, which are mainly reflected in the matching of gas path control and optimal diagnosis scheme of the gas turbine [7]. The development of construction and management mode of the gas turbine fault diagnosis and control system and the awareness and attention of the underlying technology of gas turbine monitoring system should be enhanced [8]. In order to further improve the automation effect of gas turbines in the fault diagnosis process, Wassinger et al. proposed an improved multiangle diagnosis model to judge key nodes from the common gas path composition rules [9]. Bento and Marques Cardoso made innovations in the judgment and diagnosis schemes of gas turbine fault diagnosis and proposed a semiautomatic online fault diagnosis method, which can be achieved with the help of 5G technology remote detection which has a certain application value [10]. Wang et al. analyzed different types of gas path processes from the level of gas turbine coupling analysis and proposed a fault diagnosis method based on abnormal gas path feedback mode. This method can provide the best solution according to the characteristics of the gas turbine scheme [11]. According to the different types of gas turbines, Cui et al. used different modes of differentiation methods to classify the types of gas path faults and then analyzed their differences to perform fault diagnosis [12]. In order to reduce the error rate of the gas turbine in the gas path fault diagnosis process, Han et al. adopted a multifactor diagnosis docking model and designed a verification test, which confirmed the stability and reliability of the model [13]. According to the characteristics of the working process of gas turbines, Ma et al. improved the gas path fault diagnosis strategy and proposed an ultrahigh frequency intelligent decomposition diagnosis method [14]. Vazquez-Canteli and Nagy proposed a diagnosis model based on the firefly tracing algorithm according to the specific gas turbine gas path fault diagnosis law. This model has the advantages of strong stability and good reliability [15]. Yang et al., based on the uniqueness of different types of gas turbines, developed gas path fault diagnosis strategies. This method can quickly diagnose common gas path faults according to the type of the gas turbine [16]. Research by Ayachi et al. has shown that different types of gas path diagnosis strategies can be used for gas turbines according to their differences so that the type of the gas turbine can be quickly distinguished, and the common gas path faults of this type of machinery and equipment can be from point to point; analyze formally and complete the signal conversion of the test result data and output the final diagnosis plan [17]. In order to solve the problems of low efficiency and slow data query speed of the gas turbine in group cooperation, Bibault et al. proposed a gas turbine automatic fault diagnosis and control method [18]. Shlomi et al. have constructed the efficiency evaluation basis in the gas path automatic diagnosis scheme of the gas turbine. Experiments show that the diagnosis strategy can effectively improve the gas path fault diagnosis efficiency of different gas turbines and effectively solve the problem of low accuracy in gas path control of the gas turbine by improving the cooperative work efficiency [19]. In summary, in the existing research results, most of the innovations are still focused on the matching analysis of gas turbine type judgment and gas path fault diagnosis, and intelligent analysis algorithms are not applied to many research results [20]. On the contrary, there are few research studies on the intelligent analysis of data in the process of gas turbine gas path fault diagnosis [21].

Under this background, this paper proposes an application model of intelligent fault diagnosis for the gas turbine based on reinforcement learning algorithm. The data mining technology and reinforcement learning algorithm are used in the gas path fault intelligent diagnosis scheme of the gas turbine. It can make full use of the characteristic information in different gas turbine parameter databases to realize the unified adaptive management of the gas turbine; the reinforcement learning control factor is used to quantitatively describe the degree of similarity between the comparison columns (gas path diagnosis data at different stages) and the reference columns (effective information source through preliminary screening) and the degree of agreement between the expected indicators (expected control data), so as to complete the weight ranking of influencing factors of gas turbine gas path fault intelligent diagnosis by quantitative indicators, and it can efficiently realize the adaptive diagnosis of gas path fault through different fault diagnosis control methods.

In this paper, the gas path fault intelligent diagnosis model of the gas turbine based on reinforcement learning algorithm is studied, which is mainly divided into four parts.  Section 1 introduces the research status of gas turbine fault diagnosis.  Section 2 introduces the application of reinforcement learning algorithm in gas path fault diagnosis. In Section 3, based on the fault diagnosis control system of gas turbine and common gas path fault data information, an intelligent gas path fault diagnosis model of the gas turbine based on reinforcement learning algorithm is constructed. In Section 4, the practical application effect of the gas path fault intelligent diagnosis model of the gas turbine constructed in this paper is tested, and the practicability of the intelligent diagnosis model is objectively evaluated by designing experiments and using different evaluation indexes.

## 2. The Application of Reinforcement Learning Algorithm in Gas Path Fault Intelligent Diagnosis of Gas Turbine

Reinforcement learning algorithm (deep learning algorithm) has important applications in intelligent cloud computing and other fields [22]. Common reinforcement learning technology for different types of data and information cluster, based on specific judgment index, after many times of adaptive deep learning, obtains the optimal solution or data results [23]. In the process of fault diagnosis and control of gas turbine, different types of reinforcement learning algorithms need to be selected for accurate optimal control, and the more common one is neural network algorithm [24]. Neural network algorithm, such as other greedy optimization algorithms, is a general optimization algorithm [25–30]. At present, neural network algorithm is widely used in the fault diagnosis process and control link in the field of automation. Most of the control systems with good application effect in the automatic control link of process are based on algorithm. The advantage of strong neural network algorithm in gas path fault intelligent diagnosis of the gas turbine lies in providing effective approximate solution algorithm for NLP complex problems and overcoming the dependence on the initial value. The parameters of reinforcement learning algorithm in the application process are shown in Table 1.

Based on the idea of reinforcement learning algorithm, in the process of building the gas path fault intelligent diagnosis scheme of the gas turbine, this paper selects the local adaptive neural network algorithm and designs a gas path fault monitoring model with high intelligence. Reinforcement learning algorithm is used for intelligent analysis to realize automatic fault diagnosis control and information feedback.

## 3. Intelligent Fault Diagnosis Model of Gas Turbine Based on Reinforcement Learning Algorithm

### 3.1. Monitoring and Optimization Process of Reinforcement Learning Algorithm in Gas Path Fault Intelligent Diagnosis of Gas Turbine

Gas turbine is an internal combustion-type power machine that drives the impeller to rotate at a high speed with a continuous flow of gas as the working medium and converts the energy of the fuel into useful work. It is a rotating impeller heat engine. The gas turbine has the simplest structure and can best reflect a series of advantages such as small size, light weight, fast start-up, less use, or no need for cooling water that are unique to gas turbines. According to the purpose, it can be divided into three categories: turbine engines for aviation, gas turbines used as the main propulsion power device on ships, and gas turbines for power plants on land power plants. The common fault occurrence links include electrical systems, rotor blades, pitch systems, hydraulic systems, control systems, and gearboxes. The common failure types include press surge, ignition failure, combustion failure, high lubricating oil temperature, and bending of the main shaft of the gas turbine. The sensor pattern is shown in Figure 1.

After determining the common gas path fault types of gas turbine, it is necessary to analyze the overall monitoring optimization process. Based on this, this study needs to use reinforcement learning algorithm for deep learning when analyzing different types of gas path fault data. This process requires a large number of fault data for self-learning. The specific working process is shown in Figure 2.

The deep learning process of the reinforcement learning algorithm is to group the data information in the fault diagnosis process of the gas turbine, then merge it according to its specific array, then perform the data difference amplification processing according to the common point so that it can quickly complete the classification of the array, and then combine the eigenvalue function and the control function to make further judgments, and its eigenvalue function *E*(*x*) is as follows:

(1) $$\begin{array}{c} E\left(x\right)=\sum_{i=1}^{m}\left({\left(\frac{x}{x-1}\right)}^{2}+\underset{i=1}{\sum }\sqrt{\frac{x^{2}}{m-1}}\right), \end{array}$$

where *x* is the gas path fault data and *m* is the upper limit of fault data type.

Therefore, the actual working process of reinforcement learning algorithm can be regarded as the optimization control process of repeated decreasing control parameters. When the reinforcement learning algorithm deeply mines the types of fault diagnosis, it will select the feature recognition function *Z*(*x*) for discrimination, and its expression is as follows:

(2) $$\begin{array}{c} Z\left(x\right)=\sum_{i=1}^{m}\left({\left(x^{3}+x+5\right)}^{2}+\underset{i=1}{\sum }\left(x+2\right)\sqrt{\frac{x^{2}}{x+1}}\right), \end{array}$$

where *x* is the gas path fault data and *m* is the upper limit of fault data type. In this process, the feature recognition function needs to be used to calculate the data group to be processed, and the calculated value is analyzed and judged. When the judgment result is qualified, it will be included in the normal database system; otherwise, it will continue to the fault diagnosis data which are subjected to reinforcement learning calculations until the requirements are met. The process of fault data processing in this link is shown in Figure 3.

Intelligent fault diagnosis of the gas turbine is to control and classify the fault diagnosis process of multiple gas turbines. Reinforcement learning algorithm based on neural network strategy in the actual automatic control process of gas path fault diagnosis, multidimensional cyclic calculation of gas turbine data information, when the requirements are met, and two-dimensional comparison is performed, otherwise continuously updated. The process of this link is shown in Figure 4.

According to the commonly used learning function *F*_*n*_^*m*^(*y*) and judgment function *W*_*n*_^*m*^(*y*) in reinforcement learning algorithm, we learn the gas path fault intelligent diagnosis process of the gas turbine. The expressions of learning function *F*_*n*_^*m*^(*y*) and judgment function *W*_*n*_^*m*^(*y*) are as follows:

(3) $$\begin{array}{c} F_{n}^{m}\left(y\right)=\frac{\sum_{i=1}^{m}\left({yy-1}^{2}+\sum_{i=1}\sqrt{y^{2}/y-1}\right)}{m}+\frac{\sum_{i=1}^{n}\left(y^{2}+\sum_{i=1}\sqrt{y/y-1}\right)}{n},\\ W_{n}^{m}\left(y\right)=\frac{\sum_{i=1}^{m}\sqrt{y^{2}/y-1}}{m}+\frac{\sum_{i=1}^{n}\sqrt{y/y-1}}{n}. \end{array}$$

It can be seen from the above formula that when *m* and *n* are large, the smaller the function value of *F*_*n*_^*m*^(*y*) is, the larger the function value of *W*_*n*_^*m*^(*y*) is, indicating that the control effect of *m* and *n* on the fault diagnosis process is better.

## 4. Implementation Steps of Gas Path Fault Diagnosis and Monitoring Optimization Model for Gas Turbine

After analyzing the optimization process of the scheduling algorithm of the fault diagnosis control link of the gas turbine, it is necessary to analyze and plan the overall power station monitoring process. Based on the three core steps of reinforcement learning algorithm strategy, this study analyzes the monitoring process of the gas path fault diagnosis model of the gas turbine from three dimensions. The information needed in the diagnosis process is shown in Table 2.

The first aspect is to determine the types of control parameters for different types of fault diagnosis requirements analysis process. The most important feature and advantage of the gas turbine gas path fault diagnosis and monitoring optimization model described in this research based on the reinforcement learning algorithm lie in the diagnosis of different types of faults, through the multidimensional analysis of the diagnosed gas path fault data and the secondary data cross learning, In this way, the best solution diagnosis plan can be drawn according to the difference of the gas path fault diagnosis. Diagnosis of gas path faults and the corresponding threshold function *C*(*x*) is as follows:

(4) $$\begin{array}{c} C\left(x\right)=\frac{1}{m}\sum_{i=1}^{m}{\left(x_{i}-\bar{x}\right)}^{T}w_{i}\left(x_{i}-\bar{x}\right), \end{array}$$

where *x* is the data to be diagnosed, *m* is the diagnostic extremum, and *w*_*i*_ is the threshold vector. In different scenarios, the requirement analysis process will automatically tend to the best analysis state, while the scheduling control process of the fault diagnosis process in this reinforcement learning algorithm is to find the gas path state data corresponding to the minimum value of the function (that is, the minimum time required for gas path fault diagnosis, the minimum error rate, and other reference values). So, to determine different types of the fault diagnosis scheme, the initial diagnosis process of gas path fault of the gas turbine is shown in Figure 5. It can be seen from Figure 5 that, in the single fault diagnosis simulation process, the amount of fault diagnosis has good stability, and as the number of diagnoses increases, the number of faults diagnosed gradually becomes stable. This is because as the number of fault diagnosis increases, the number of faults gradually tends to the upper limit bottleneck stage, and each iteration of fault diagnosis will increase and will not be eliminated, so the number of faults diagnosed gradually tends to smoothing (that is, gradually approaching the upper limit of real failures).

Secondly, the accuracy of control parameters in different types of fault diagnosis planning is determined. In the process of determining the fault diagnosis plan of the gas turbine intelligent diagnosis model described in this article, the reinforcement learning algorithm used is analyzed based on different types of data. In real-time and accurate judgment of different fault diagnosis data, through iterative processing of the vector data corresponding to the fault diagnosis correlation data information represented by each gas turbine data, a standardized gas path fault diagnosis scheduling is realized. The vector represented by the plan is the basic criterion, and its precision control function *d*_Δ_(*x*_1_, *x*_2_) is as follows:

(5) $$\begin{array}{c} d_{\Delta }\left(x_{1},x_{2}\right)={\left(\max\left(r_{1},r_{2}\right)-\overset{r_{1},r_{2}}{\underset{i,j=1}{\sum }}{\left(x_{1,i}^{T}x_{2,j}\right)}^{2}\right)}^{1/2}, \end{array}$$

where *x* is the data to be diagnosed and *r* is the reference extremum, and then, the differences are compared according to the monitoring thresholds of different gas path types of the gas turbine, so as to improve the adaptive efficiency and accuracy of the gas turbine in the fault diagnosis process.

Thirdly, the type and range of the key antidisturbance coefficient of the gas turbine in gas path fault diagnosis are determined. Reinforcement learning algorithm begins to play its role in data analysis for the gas path fault diagnosis device and the overall monitoring scheme of the gas turbine, After several times of optimization of the fault diagnosis scheduling scheme of this cycle, the monitoring and optimization process of the whole gas turbine will be realized according to the guidance of the scheme. The optimization function *T*(*x*) is as follows:

(6) $$\begin{array}{c} T\left(x\right)={\sum_{j=1}^{n}\mu \left(\frac{x_{j}}{n}-d_{ij}\right)}^{2}. \end{array}$$

Among them, *x* is the data to be diagnosed, *μ* is the reference coefficient, *n* is the type limit value, and *d*_*ij*_ is the standard degree.

In order to obtain a solution set suitable for the current state according to its different conditions, the optimal value index of reinforcement learning algorithm is used to classify and evaluate the diagnosis efficiency and control failure rate of different fault diagnosis scheduling processes. Then, the fault diagnosis data information of the core database commonly used in the automatic diagnosis and control system in the gas turbine is controlled and monitored for the second time. Then, the stability and efficiency of the gas turbine monitoring model based on adaptive reinforcement learning control strategy and neural network technology are guaranteed. The whole process of fault diagnosis and judgment is shown in Figure 6. It can be seen from Figure 6 that, during the fault diagnosis process, as the diagnosis completion degree increases, the diagnosis results also show a gradual increase rule, and as the diagnosis completion degree exceeds 90%, the fault diagnosis is quantified. The characterization index has increased significantly because with the increase of the degree of completion of diagnosis, more types of faults have been completed in a shorter period of time.

## 5. Result Analysis and Discussion

### 5.1. Experimental Test Process of Gas Path Fault Diagnosis Control Model of Gas Turbine

After the establishment of gas turbine monitoring optimization model based on reinforcement learning algorithm, it is necessary to verify its scientificity in practice. In order to ensure the authenticity and randomness of the experiment, the industry general experimental indicators are used to set the experiment. The reference experimental standards are shown in Table 3.

During the experiment, the initial results of five groups of experimental data are shown in Figure 7.

In the reliability analysis of the experimental results, the reliability is divided into 8 levels from 1 to 8. The horizontal axis represents the number of diagnoses during the experiment, and the vertical axis represents the quantitative reference value of the reliability of the diagnosis result. The higher the level, the better the reliability. It can be seen from Figure 6 that the reinforcement learning optimization model is more reliable than the other four methods, and the number of faults diagnosed is also the largest. This is because when analyzing different types of gas path fault data, it will pass the reinforcement learning strategy, realizes the rapid fusion analysis of the fault information in the gas turbine, and also uses the data generated by the gas turbine fault diagnosis control process and other characteristic information (such as the loss of the gas turbine gas path fault intelligent diagnosis process, control efficiency, and accuracy), to further obtain the data feedback of the gas turbine monitoring model's behavior during the entire optimization control process, to achieve substantial control efficiency improvement, and to realize the multidimensional monitoring analysis and program planning of the gas turbine. In this way, high-precision and high-efficiency query can be achieved so that, under the gas turbine monitoring model, accurate program planning for different types of fault diagnosis data in the gas path of each gas turbine can be achieved.

### 5.2. Experimental Results and Analysis

According to the intelligent model proposed in this study, by observing the experimental data of the gas turbine monitoring model based on reinforcement learning algorithm, the reinforcement learning stability results are shown in Figure 8 (5 points), the horizontal axis is the number of diagnosed test results, and the vertical axis is the stability index of reinforcement learning.

According to the results in Figure 7, compared with the traditional gas path fault intelligent diagnosis model, the data stability of the gas path fault intelligent diagnosis model based on reinforcement learning algorithm is greatly improved (the stability performance reaches the limit score of 5 in the fifth round) and shows a relatively stable trend. This shows that the proposed model has better applicability. The error of the experimental results is shown in Table 4, the traditional data processing model refers to the current mainstream nonlinear data processing model (error analysis based on multivariate functions), and the single neural network model refers to the data processing model that only uses neural networks without reinforcement learning.

It can be seen from Table 4 that, in terms of error control, the error rate of the gas turbine monitoring model based on reinforcement learning algorithm is lower, only 2.09%, which is significantly smaller than the results of the other two methods. In addition, gas turbine groups with different data eigenvalues of different groups can be adaptively and accurately controlled by the monitoring system, and other differences can be well distinguished to achieve steady-state regulation. This shows that the gas path fault intelligent diagnosis model of the gas turbine based on reinforcement learning algorithm can distinguish the differences of different types of gas path fault diagnosis, to realize the control of any gas path fault intelligent diagnosis link of the gas turbine.

## 6. Conclusion

There are some problems in the application of the common intelligent fault diagnosis scheme of the gas turbine in China. Based on this, this paper studies the gas path fault intelligent diagnosis model of the gas turbine based on reinforcement learning algorithm. Firstly, a gas path fault diagnosis and monitoring model with strong adaptability is designed to realize the unified management of different types of gas path fault data sources. According to the data differences in the process of fault diagnosis, reinforcement learning algorithm is used for intelligent analysis. The intelligent generation of gas path fault diagnosis scheme for the gas turbine is realized. Secondly, the reinforcement learning algorithm is applied in the gas path fault diagnosis, making full use of the information source in the gas turbine database to realize the unified monitoring, planning, and management of the gas turbine in the gas path fault diagnosis. Finally, the experimental results show that the gas path fault intelligent diagnosis model based on reinforcement learning has better performance stability and lower error. However, this study only considers the control accuracy and diagnosis efficiency and does not consider the cost optimization. Therefore, further research can be carried out from the cost of gas path fault diagnosis of the gas turbine.

## Figures and Tables

**Figure 1:** Sensor graphics.

**Figure 2:** The working process of the reinforcement learning algorithm.

**Figure 3:** Data processing process for faults.

**Figure 4:** Fault diagnosis process of gas turbine gas path based on feedback strategy.

**Figure 5:** The first diagnosis process of gas turbine's gas path breakdown.

**Figure 6:** The overall fault diagnosis and judgment process.

**Figure 7:** Initial results of 5 sets of experimental data.

**Figure 8:** Reinforcement learning stability of experimental results.

**Table 1:** Parameters that need to be set during the application of the reinforcement learning algorithm.

Set indicator	Common reference value
Number of sample reference categories	100
Value function setting number	30
Number of learning gradients	37
Number of learning layers	46

**Table 2:** Information needed during diagnosis.

Information type	The first stage	The second stage	The third phase
Data reliability	0.9	0.95	0.98
Reinforcement learning times	5	10	15
Data analysis times	4	9	14

**Table 3:** Statistical data reference value of gas path fault diagnosis experiment.

Air circuit failure index	Pneumatic fault reference value
Number of samples	4000
Characteristic number	3596
Accuracy	0.95
Number of categories	30
Domain representation	18
Reinforcement learning type	Strategy-centered and step-by-step reinforcement learning
Fault diagnosis model	Press surge, ignition failure, combustion failure, high lubricating oil temperature and bending of the main shaft of the gas turbine, etc.
Number of neural network layers	33
Number of neural network nodes	107

**Table 4:** Error of experimental results.

Error of experimental results	Error percentage (%)
Reinforcement learning model	2.09
Traditional data processing model	3.19
Single neural network model	3.15

## Data Availability

The data used to support the findings of this study are available from the corresponding author upon request.
